# The Value of 18F-FDG PET/CT in the Diagnosis of Tuberculous Pleurisy and in the Differential Diagnosis between Tuberculous Pleurisy and Pleural Metastasis from Lung Adenocarcinoma

**DOI:** 10.1155/2022/4082291

**Published:** 2022-07-31

**Authors:** Xiaoqing Du, Feng Zhu, Chunjing Yu

**Affiliations:** ^1^Nuclear Medicine Department of the Affiliated Hospital of Jiangnan University, Wuxi, China; ^2^Respiratory Medicine Department of the Fifth People's Hospital of Wuxi (Infectious Disease Hospital of Wuxi), Wuxi, China

## Abstract

**Objectives:**

This study aims to investigate the diagnostic value of 18F-FDG PET/CT in tuberculous pleurisy (TBP) and the differential diagnostic value of 18F-FDG PET/CT between TBP and pleural metastasis from lung adenocarcinoma (PMLAC).

**Materials and Methods:**

The features of pleura on PET and hybrid CT were retrospectively studied in 20 patients with TBP and 32 patients with PMLAC. The ROC curve was used to evaluate the diagnostic effectiveness of these indices for TBP and PMLAC, and binary logistic regression analysis was conducted to identify independent predictors of TBP and PMLAC.

**Results:**

There were significant differences in pleural 18F-FDG uptake pattern on PET (*P*=0.001), pleural morphology pattern on CT (*P*=0.002), the maximum diameter of the pleural nodule (*P*=0.001), and interlobular fissure nodule (*P*=0.001) between TBP and PMLAC groups. The diffused pleural FDG uptake type on PET (odds ratio (OR) = 6.0, 95% CI 2.216–16.248, *P*=0.001) and the lamellar pleural thickening type on CT (OR = 4.4, 95% CI 2.536–7.635, *P*=0.001) were independent predictors of TBP, with 60% and 55% sensitivity, 96.6% and 90.6% specificity, and 82.7% and 77.0% accuracy. The combined diagnostic sensitivity, specificity, and accuracy for TBP were 70%, 87.5%, and 80.8%. The mixed pleural FDG uptake type on PET (OR = 5.106, 95% CI 2.024–12.879, *P*=0.001), the mixed pleural thickening type on CT (OR = 2.289, 95% CI 1.442–3.634, *P*=0.001), and the maximum diameter of the pleural nodule (OR = 1.027, 95% CI 1.012–1.042, *P*=0.001) were independent predictors of PMLAC, with 78.1%, 71.9%, and 87.5% sensitivity, 85%, 80%, and 85% specificity, and 80.8%, 75%, and 86.5% accuracy. The combined diagnostic sensitivity, specificity, and accuracy for PMLAC were 96.9%, 85%, and 90.4%.

**Conclusions:**

18F-FDG PET/CT is of great clinical value in the diagnosis of TBP and in the differential diagnosis between TBP and PMLAC.

## 1. Introduction

Tuberculosis (TB) is a communicable disease, that is a major cause of illness, one of the top 10 causes of death worldwide, and the leading cause of death from a single infectious agent. The disease typically affects the lung (pulmonary TB) but can also affect other sites (extrapulmonary TB). Extrapulmonary TB represented 16% of the 7.1 million incident cases that were notified in 2019 [1]. It affects the lymph node most frequently, followed by pleural infection [2]. The incidence of pleural involvement in TB nonendemic areas is 3–5% [3], whereas it approaches 30% in TB endemic areas [4].

Previous studies have used 18F-FDG PET/CT to detect TB and assess disease activity as well as the extent of the disease. By far, few studies focusing on 18F-FDG PET/CT in TBP have been published, but there was no study on 18F-FDG PET/CT in distinguishing TBP from PMLAC. In this study, we attempt to investigate the diagnostic value of 18F-FDG PET/CT for TBP and the differential diagnostic value between TBP and PMLAC for the first time.

## 2. Materials and Methods

### 2.1. Study Base

All patients who underwent 18F-FDG PET/CT for nonreason pleural effusion between January 2010 and September 2021 at the nuclear medicine department of the Affiliated Hospital of Jiangnan University (Wuxi, China) were evaluated retrospectively. The study protocol was approved by the institutional review board and ethics committee. Patients' informed consent was waived because of the retrospective nature of the study design.

Inclusion criteria were as follows: (1) with unexplained pleural effusion as the first symptom; (2) exudate was defined according to Light's criteria; (3) no history of tumor; (4) definitive diagnosis supported by final pathology or follow-up result.

Confirmative diagnostic criteria of TBP were as follows: (1) *Mycobacterium tuberculosis* (*Mtb*) was found in the sputum, pleural effusion, or pleural biopsy specimen; (2) a positive TB culture of the sputum or pleural fluid; (3) demonstration of caseated granuloma in the pleural biopsy specimen; (4) evidence of clinical improvement after antituberculosis chemotherapy.

Malignant effusion was diagnosed if a malignant cell was found in the cytological examination of the pleural effusion or in the pleural biopsy specimen. According to the purpose of this study, only LAC-associated malignant effusion was enrolled.

### 2.2. PET/CT Acquisition and Image Analysis

A total of 52 patients matched the inclusion criteria. All patients were required to fast for at least 6 h before 18F-FDG (5.55 MBq/kg) intravenous injection. Acquisition was conducted 60 min after the injection. The patient was placed in a supine position on the scanner bed. Imaging data were acquired from the skull to the thigh at a 1.5 min/bed position. Low-dose CT was performed for attenuation correction and lesion localization.

All patients with PMLAC received high-resolution thin-layer chest CT at maximum inspiration by using the same machine after the routine PET/CT scan, with 120 kVp, 140 mAs, and a pitch of 1.2. The image was reconstructed using a medium sharp reconstruction algorithm with a thickness of 1 mm. The CT image was photographed using a window level of −600 HU and a window width of 1200 HU for the lung window.

Regions of interest (ROIs) were drawn manually on the lesion sites based on the corresponding CT images.

The PET/CT Scanner was from Siemens (Biograph True Point PET/CT). Two physicians evaluated the images independently, and discrepancies were resolved by consultation.

### 2.3. Visual Analysis

Visual analysis mainly focused on the morphology of the pleura on PET and CT, respectively, and whether there were abnormal lesions in the lung.

Pleural FDG uptake patterns on PET were classified into four types: (1) no FDG uptake; (2) focal FDG uptake; (3) diffused FDG uptake; (4) mixed FDG uptake meaning coexistence of focal uptake and diffused uptake.

The pleural morphologies on CT were classified into four patterns: (1) normal pleura; (2) nodule formation; (3) lamellar thickening; (4) mixed thickening meaning coexistence of nodule formation and lamellar thickening. Maximum diameters of pleural nodules were measured on CT. All data units of length were expressed in centimeters.

The distance between LAC and pleura and the morphology of interlobular fissure on high-resolution thin-layer chest CT in the PMLAC group were observed.

### 2.4. Semiquantitative Analysis and Quantitative Analysis

The highest SUVmax and lowest SUVmax of pleural lesions, SUVmax of interlobular fissure nodules, and SUVmax of LAC lesions were measured on PET images.

Maximum diameters of pleural nodules and interlobular fissure nodules and maximum diameters as well as minimum diameters of LAC lesions were recorded.

### 2.5. Laboratory Examination

The T-cell enzyme-linked immune spot test (T-SPOT) of venous blood and adenosine deaminase (ADA) value of effusion in the TBP group within 2 weeks before the PET/CT scan were collected.

### 2.6. Statistical Analysis

Data were analyzed using SPSS Statistics 23.0. Continuous variables with normal distribution were expressed as the mean ± standard deviation, and continuous variables without normal distribution were expressed as median and interquartile range. Differences between the two groups were analyzed by the independent-sample *t*-test or Mann–Whitney *U* test. The Spearman test was used to analyze the correlation ship, and binary logistic regression analysis was used to identify independent predictors. The receiver operating characteristic (ROC) curve was used to analyze the diagnostic value. *P* < 0.05 denoted statistical significance.

## 3. Results

### 3.1. Patient Characteristics

A total of 52 patients were enrolled, including 20 patients with TBP and 32 patients with PMLAC. The clinical characteristics of each group are summarized in Table 1. Positive rates of night sweat and fever (ranging from 37.5–39.5°C) in patients with TBP were 20% (4/20) and 40% (8/20), whereas no patient with PMLAC presented these symptoms. The positive rate of chest pain in patients with PMLAC was 18.75% (6/32), whereas no patient with TBP presented this symptom.

### 3.2. TBP Group

A total of 20 patients with TBP were enrolled in this study. The positive rate of TB history was 25% (5/20), including 4 patients with lung TB history and 1 patient with renal TB history, and the longest time interval was 50y. The positive rate of cases presenting active TB lesions in other organs was 70% (14/20), including 9 patients with lung TB, 3 patients with peritoneum TB, 1 patient with ilium TB, and 1 patient with brain TB. Acid-fast bacilli were found in sputum smears in 20% (4/20) of cases, and sputum cultures were positive in 10% (2/20) of cases, all of these accompanied by active lung TB. The positive rate of T-SPOT was 40% (8/20). ADA values of pleural effusions were obtained in 16 of 20 patients with TBP. The pleural effusion ADA value was 23.33 ± 19.52, and the positive rate of that was 56.25% (9/16).

Twelve cases presented diffused pleural FDG uptake type on PET (Figure 1), 3 presented focal type, 3 presented mixed type, and 2 showed no FDG uptake (Figure 2). SUVmax of the highest pleural uptake lesion and the lowest pleural uptake lesion was 6.11 ± 4.03 and 1.88 ± 1.22.

Eleven cases presented lamellar pleural thickening on CT (Figure 1), 4 presented mixed thickening, 4 showed no obvious changes of pleura (Figure 2), and 1 presented nodule formation. The maximum diameter of pleural nodules in TBP group was 0.0 (0.0, 0.0).

### 3.3. PMLAC Group

A total of 32 patients with PMLAC confirmed by pathology were included in this study.

Twenty-five cases presented mixed pleural FDG uptake type on PET (Figure 3), 5 presented focal type, 1 presented diffused type, and 1 showed no FDG uptake. SUVmax of the highest uptake lesion and the lowest uptake lesion of the pleura was 4.55 (3.25, 7.05) and 1.73 ± 0.87.

Twenty-three cases presented mixed pleural thickening on CT (Figure 3), 5 presented nodule formation, 3 presented lamellar thickening, and 1 showed no obvious change of pleura on CT.

About 78.12% (25/32) of LAC lesions were discovered on PET/CT, whereas 21.88% (7/32) of LAC lesions were undiscovered on PET/CT. Maximum and minimum diameters of LAC lesions were 2.84 (1.65, 4.20) and 1.84 (1.29, 2.79). The SUVmax of LAC lesions was 10.29 ± 5.44. The maximum diameter of pleural nodules was 1.0 (0.75, 1.27).

LAC with a pleural indentation or pleural attachment (no visible space between the LAC lesion and pleura on CT images at the lung window), shown on high-resolution thin-layer chest CT at maximum inspiration, was visible in all 25 PMLAC patients.

Interlobar fissure nodules were found in 68.8% (22/32) of patients with PMLAC (Figure 4) but none in patients with TBP. The maximum diameter of the interlobular fissure nodule was 0.90 ± 0.34, and the SUVmax was 2 ± 2.30.

### 3.4. Comparison between the TB Group and PMLAC Group

There were significant differences in night sweat (*P*=0.029), fever (*P*=0.001), chest pain (*P*=0.041), pleural FDG uptake type on PET (*P*=0.001), pleural morphology on CT (*P*=0.002), the maximum diameter of the pleural nodule (*P*=0.001), and interlobular fissure nodule (*P*=0.001) between TBP and PMLAC groups. There were no significant differences in age, sex, other symptoms, and SUVmax of pleural lesions between the two groups.

### 3.5. A Correlation Study Demonstrated a Significant Correlation between the Interlobular Fissure Nodule (*r* = 0.677, *P* = 0.001) and PMLAC

Binary logistic regression analyses identified the diffused pleural FDG uptake type on PET (OR = 6.0, 95% CI 2.216–16.248, *P*=0.001) and the lamellar pleural thickening type on CT (OR = 4.4, 95% CI 2.536–7.635, *P*=0.001) were independent predictors of TBP, with areas under ROC curves of 0.784 and 0.728, with 60% and 55% sensitivity, 96.6% and 90.6% specificity, and 82.7% and 77.0% accuracy. When combined with the diffused pleural FDG uptake type on PET and the lamellar pleural thickening type on CT, the area under the ROC curve was 0.821, with 70% sensitivity, 87.5% specificity, and 80.8% accuracy.

The mixed pleural FDG uptake type on PET (OR = 5.106, 95% CI 2.024–12.879, *P*=0.001), the mixed pleural thickening type on CT (OR = 2.289, 95% CI 1.442–3.634, *P*=0.001), and the maximum diameter of the pleural nodule (OR = 1.027, 95% CI 1.012–1.042, *P*=0.001) were independent predictors of PMLAC, with areas under ROC curves of 0.816, 0.759, and 0.838, with 78.1%, 71.9%, and 87.5% sensitivity, 85%, 80%, and 85% specificity, and 80.8%, 75%, and 86.5% accuracy. The optimal diagnostic cut-off value of the maximum diameter of the pleural nodule was 0.425. When combined with the mixed pleural FDG uptake type on PET and the mixed pleural thickening type on CT, the area under the ROC curve was 0.827, with 84.4% sensitivity, 80% specificity, and 84.6% accuracy. When combined with the mixed pleural FDG uptake type on PET, the mixed pleural thickening type on CT, and the maximum diameter of the pleural nodule, the area under the ROC curve was 0.878, with 96.9% sensitivity, 85% specificity, and 90.4% accuracy. The area under the ROC curve of the interlobular fissure nodule was 0.844, with 68.8% sensitivity, 100% specificity, and 80.8% accuracy.

## 4. Discussion

*Mtb* is an aerobic, obligate intracellular microorganism that features an unusually complex and thick cell wall that is impermeable to several compounds [5]. When a patient is infected with *Mtb*, the cell-mediated immunity of the host results in either clearing of the infection or the restriction of bacilli inside granulomas giving rise to a latent TB infection (LTBI). LTBI state might last for the entire life span of the individual or progress to active TB by reactivation of the existing infection with a lifetime risk of 5–10% [6]. Up to 25% of patients with TBP had TB history in this study, the longest time interval was 50y, and all had received up to 6 months of therapy before. We assumed that *Mtb* in these patients had not been eliminated after previous therapy and had converted to latency, waiting for the proper time to multiply again and reach the pleura through blood.

Pleural effusion is a common clinical problem, which can be caused by >50 diseases [7]. TBP is one of the most frequent causes of pleural exudate globally [2]. In China, TBP accounts for about 25% of all TB cases [8]. Classic features of TB include chronic cough, weight loss, fever, night sweat, and hemoptysis. The number of patients with night sweat and fever in the TBP group was significantly higher than that in the PMLAC group in this study, while the number of patients with chest pain in the PMLAC group was significantly higher than that in the TBP group.

To date, the diagnosis of TBP remains a challenge. The conclusive diagnosis of TBP depends upon the isolation of *Mtb* from sputum, pleural fluid, or pleural biopsy specimens. The positive rate of sputum acid-fast bacilli smear is 12%, and the sensitivity of pleural fluid culture is <40% [2, 7]. The positive rate of sputum acid-fast bacilli was 20% in this study, higher than the previous ones, which may be caused by the high proportion of patients with concurrent pulmonary TB. The positive rate of sputum culture was 10% in this study.

T-SPOT is based on the detection of the interferon-gamma (IFN-*γ*) cytokine. Some previous studies reported that certain bacteria(*Mycobacterium kansasii*, *Mycobacterium szulgai*, and *Mycobacterium marinum*), hematologic malignancies, and empyema can cause false positive in T-SPOT via the stimulation of IFN-*γ* secretion [9, 10]. The positive rate of T-SPOT in peripheral blood was 40% in this study. Numerous studies suggested that ADA was one of the more reliable and cost-effective pleural fluid biomarkers of TBP [11, 12]. The normal reference range of the pleural effusion ADA level in our laboratory is 4–24 U/L. The pleural effusion ADA value was 18.95 (0.45, 39.68) in this study, and the positive rate of that was 56.25%. ADA is also a nonspecific inflammatory and immune response marker for TB, such as higher false-negative rates in individuals with liver cirrhosis or HIV infection and false-positive rates in patients with malignancy-related fluid, bacterial pneumonia or pulmonary empyema, and rheumatoid arthritis [2].

TB lesions contain many epithelioid cells, lymphocytes, and Langerhans cells that have a high expression of glucose transporter 1 (Glut-1) and Glut-3, which induce high 18F-FDG uptake [13]. 18F-FDG PET/CT can play an important role in TB patients' management, particularly for those whose sputum smear and sputum culture are negative, unable to produce sputum, or have EPTB [14, 15].

Visual thoracoscope diagnosis of TBP is based on the presence of multiple yellowish-white miliary tubercles of uniform size (usually < 5 mm) on the visceral and parietal pleura. Although these multiple miliary nodules can be detected, their sizes are too small to identify their nodular features by CT, which yields a CT pattern of smooth uniform thickening [16]. Shimamoto proposed that diffused peritoneal uptake of FDG may be indicative of tuberculous peritonitis rather than peritoneal carcinomatosis and smooth uniform thickening was a significant predictor of tuberculous peritonitis, with 60% sensitivity and 92.2% specificity [17]. Other case reports also described diffused 18F-FDG uptake in the peritonea of patients with tuberculous peritonitis [18, 19]. The diffused pleural FDG uptake type on PET and the lamellar pleural thickening type on CT were independent predictors of TBP in this study, with 60% and 55% sensitivity, 96.6% and 90.6% specificity, and 82.7% and 77.0% accuracy. When combined with the diffused pleural FDG uptake type on PET and the lamellar pleural thickening type on CT, the area under the ROC curve was 0.821, with 70% sensitivity, 87.5% specificity, and 80.8% accuracy.

The manifestation of TB varies depending on the immune status of the host. While high FDG uptake lesions in a patient with TB may represent an active disease, they may also represent a host immune system response that will eventually prevail [20]. As the CD4 count drops, the presentation becomes atypical, with atypical pulmonary manifestations and a greater proportion of patients (>50% in some cases) presenting with EPTB. At very low CD4 counts, the pulmonary features of the disease may be completely absent and disseminated TB may present as a nonspecific febrile illness with high mortality [21, 22]. One patient with TBP presented a fever of 39.5°C and showed no obvious pleural 18F-FDG uptake in this study, which was speculated to be related to the decreased function of the patient's immune system.

Previous studies using 18F-FDG PET/CT to differentiate TBP from malignant pleural or peritoneal disease mostly enrolled patients with primary malignant tumors of the pleura or peritoneum, such as malignant mesothelioma, causing most primary malignant tumors with pleura or peritoneum metastasis to be identified by CT, MRI, or 18F-FDG PET/CT, especially the primary lung malignant tumor. However, it is difficult to differentially diagnose TBP from PMLAC in some patients whose LAC lesions were undiscovered by CT or 18F-FDG PET/CT. Positive rates of discovered and undiscovered LAC lesions on 18F-FDG PET/CT in this study were 78.12% (25/32) and 21.88% (7/32). Reasons for undiscovered LAC lesions may be that LAC lesions were too small in these patients, LAC lesions were blocked by large amounts of pleural effusion, LAC lesions were too close to the pleura leading to difficulty to distinguish them from pleural metastases, or there was LAC lesion apoptosis. Accurate differential diagnoses in these patients have significant impacts on subsequent treatment.

Özmen et al. study reported that there was no significant difference in pleural SUVmax values between the malignant pleural mesothelioma (MPM) group and the TBP group [23]. Wang et al. study indicated that SUVmax did not reveal a significant difference between TBP and peritoneal carcinomatosis (PC) [24]. The result of this study was consistent with the previous ones.

A previous study reported that parietal pleural thickening greater than 1 cm was helpful in distinguishing benign cases from malignant ones [25]. Özmen et al.'s study reported that the mean pleural thickness was 21.4 ± 18.6 mm in the MPM group and 6.8 ± 3.5 mm in the TBP group [23]. The maximum diameter of the pleural nodule was 0.0 cm (0.0, 0.0) in the TBP group, whereas it was 1.0 cm (0.75, 1.27) in the PMLAC group in this study, which were consistent with the above. The optimal diagnostic cut-off value of the maximum diameter of the pleural nodule was 0.425 cm in this study.

The mixed pleural FDG uptake type on PET, the mixed pleural thickening type on CT, and the maximum diameter of the pleural nodule were independent predictors of PMLAC in this study, with 78.1%, 71.9%, and 87.5% sensitivity, 85%, 80%, and 85% specificity, and 80.8%, 75%, and 86.5% accuracy. When combined with the mixed pleural FDG uptake type on PET and the mixed pleural thickening type on CT, the area under the ROC curve was 0.827, with 84.4% sensitivity, 80% specificity, and 84.6% accuracy. When combined with the mixed pleural FDG uptake type on PET, the mixed pleural thickening type on CT, and the maximum diameter of the pleural nodule, the area under the ROC curve was 0.878, with 96.9% sensitivity, 85% specificity, and 90.4% accuracy.

Pleural indentation has been universally considered as an independent predictive factor of visceral pleural invasion (VPI) and lymphovascular invasiveness in non-small-cell lung cancer (NSCLC) [26, 27]. Some studies found that patients with a shorter distance to the visceral pleura, pleural indentation, and adenocarcinoma were more likely to have VPI [28, 29]. The maximum and minimum diameters of LAC lesions were 2.84 (1.65, 4.20) and 1.84 (1.29, 2.79) in this study. The discovered LAC lesions in this study all presented pleural indentation or pleural attachment, which was consistent with previous studies.

We found that interlobular fissure morphology presented different features in patients with TBP and PMLAC. Interlobular fissure nodules were found in 68.8% (22/32) of patients with PMLAC but none in patients with TBP. The maximum diameter of the interlobular fissure nodule was 0.90 ± 0.34, and the SUVmax was 2.57 ± 2.31. Correlation analysis identified that the interlobar fissure nodule was positively correlated with PMLAC. The area under the ROC curve of the interlobular fissure nodule was 0.844, with 68.8% sensitivity, 100% specificity, and 80.8% accuracy. We did not find an explanation for this disparity in the previously published articles. Katsuya Kato reported 55% of patients in the early MPM group with interlobular fissure irregularity, whereas no patient in the benign asbestos pleural effusion group showed this feature [30]. Yilmaz et al. reported in 1998 that of 66 patients with proven TBP, 6 (9%) were involved in the interlobular fissure, whereas the picture showed that the interlobular fissure involved in his study presented layer thickening [31]. Therefore, we believe that multiple nodular interlobular fissure changes can provide additionally important differential diagnostic value for TBP and PMLAC, especially in those patients whose LAC lesions were undiscovered by CT or 18F-FDG PET/CT.

### 4.1. Limitations

This study has some limitations. The primary limitation is that it is a retrospective study. The selection bias limitation is that the study was from a single institution and had a small sample size, which limits the extension of our findings to the general population. A large-scale study is needed in the future.

## 5. Conclusions

18F-FDG PET/CT is of great clinical value in the diagnosis of TBP and in the differential diagnosis between TBP and PMLAC. Although the SUVmax of pleural lesions showed no significant difference between the two groups, the FDG uptake pattern and CT morphology pattern of pleural lesions can provide important diagnostic information, especially for those patients whose LAC lesions were undiscovered by CT or 18F-FDG PET/CT.

## Figures and Tables

**Figure 1:** An 85-year-old man presented with cough and chest tightness and was diagnosed with TBP by thoracoscopic biopsy. (a, c, d) Diffused 18F-FDG uptake of the left pleura (red arrow). (b) Lamellar thickening of the left pleura (red arrow).

**Figure 2:** A 74-year-old man presented with chest tightness and was diagnosed with TBP by thoracoscopic biopsy. (b) Bilateral pleural effusion. (a, c, d) Normal 18F-FDG uptake of both pleurae.

**Figure 3:** A 71-year-old man presented with cough and was diagnosed with PMLAC by thoracoscopic biopsy, whose LAC lesion was undiscovered by CT or 18F-FDG PET/CT. (a) Mixed 18F-FDG uptake of the left pleura. (c, d) Diffused 18F-FDG uptake of the left pleura. (b) Lamellar thickening of the left pleura. (f, g, i, j) Focal 18F-FDG uptake of the left pleura. (e, h) Multiple nodules on the left pleura. All are indicated by the red arrow.

**Figure 4:** A 71-year-old man presented with pleural effusion and was diagnosed with PMLAC. (a, c, d, f, g) Mixed 18F-FDG uptake of the right pleura (red arrow). (b, e) Nodules on the right pleura (red arrow). (a, h–l) The primary LAC lesion of the right lung (green arrow). (l, m) Multiple nodules on the interlobular fissure (blue arrow).

**Table 1:** Characteristics of patients with TBP and PMLAC.

	Pathology	
	TBP (20)	PMLAC (32)
*Sex*		
Male	17	22
Female	3	10
Age	73.50 (62.75, 77.0)	63.59 ± 13.73

*Symptom*		
Cough	11	12
Night sweat	4	0
Fever	8	0
Hemoptysis	1	0
Feeble	2	1
Chest tightness	8	9
Asthma	2	3
Chest pain	0	6

*Visual analysis*		
No uptake	2	1
Focal uptake	3	5
Diffused uptake	12	1
Mixed uptake	3	25

*SUVmax of pleural lesions*		
SUVmax of the highest	6.11 ± 4.03	4.55 (3.25, 7.05)
SUVmax of the lowest	1.88 ± 1.22	1.73 ± 0.87

*Pleural morphology on CT*		
Normal	4	1
nodule formation	1	5
Lamellar thickening	11	3
Mixed thickening	4	23
The maximum diameter of the pleural nodule	0 (0, 0)	1.0 (0.75, 1.27)

*The interlobular fissure nodule*		
Numbers	0	22
Size	—	0.90 ± 0.34
SUVmax	—	2.57 ± 2.30

TBP: tuberculous pleurisy; PMLAC: pleural metastasis from lung adenocarcinoma.

## Data Availability

The data used to support the findings of this study are available from the corresponding author upon request.
